# Relationship between CRP Albumin Ratio and the Mortality in Critically Ill Patients with AKI: A Retrospective Observational Study

**DOI:** 10.1155/2021/9957563

**Published:** 2021-09-30

**Authors:** Jiajia Wang, Kai Zhao, Xuehui Mao, Yabin Zhang, Jing Shao, Weihua Fan, Yong Wang

**Affiliations:** ^1^Department of Clinical Laboratory, Shandong Provincial Hospital, Cheeloo College of Medicine, Shandong University, Jinan, Shandong 250021, China; ^2^Information Network Management Office, Shandong Provincial Hospital Affiliated to Shandong First Medical University, Jinan, Shandong 250021, China; ^3^Department of Gastrointestinal Surgery, Shandong Provincial Hospital Affiliated to Shandong First Medical University, Jinan, Shandong 250021, China; ^4^Department of Clinical Laboratory, Shandong Provincial Hospital Affiliated to Shandong First Medical University, Jinan, Shandong 250021, China

## Abstract

**Background:**

AKI is known to be associated with inflammation and nutritional status. The novel inflammatory prognostic score CAR (CRP/albumin ratio), which combines inflammation and nutritional status, was hypothesized to be associated with mortality in critically ill AKI patients in this study.

**Methods:**

The included cases were patients admitted to the ICU of Shandong Provincial Hospital from January 2016 to November 2018 and diagnosed with AKI within 48 hours of ICU admission. From the electronic case database of Shandong Provincial Hospital, we extracted the baseline demographic information, vital signs, routine laboratory parameters, complications, and other data. The above records are measured within 48 hours of admission to ICU. The clinical endpoint was the total cause mortality rate in hospital and 2 years. We constructed two multivariate regression models to determine the statistically significant correlation between CAR and mortality and conducted subgroup analysis to determine the mortality among different subgroups.

**Results:**

A total of 580 patients were included in this study. In multivariate regression analysis, higher CAR was associated with an increase in hospital and two-year all-cause mortality in critically ill patients with AKI after adjusting gender, age, respiratory frequency, temperature, and other confounding factors (tertile 3 versus tertile 1: OR, 95% CI: 2.97, 1.70-5.17; 3.03, 1.68-5.47, respectively; *P* < 0.001). Subgroup analysis showed that the CAR level in each subgroup increases with hospital mortality in critically ill patients with AKI.

**Conclusion:**

The increase of CAR in critically ill patients with AKI was associated with an increased risk of all-cause death.

## 1. Introduction

Acute kidney injury (AKI) is a severe clinical syndrome characterized by a rapid decline in renal function due to multiple causes with a higher incidence of morbidity and mortality, especially in patients admitted to intensive care units (ICU) [1, 2]. The incidence of AKI in patients admitted to ICU is reported to be 36%, with a higher mortality rate of 60-70% [3, 4]. Moreover, surviving patients often fail to recover renal function and require lifelong renal replacement therapy [5, 6], severely reducing their quality of life and increasing the financial burden. Given the high incidence and mortality of AKI, researchers actively investigate the various factors associated with AKI's occurrence and prognosis to take effective interventional measures to improve survival in the early stage. They have also made some achievements [7–9].

AKI is a complex disease with multiple etiologies and risk factors, usually following other acute and chronic conditions. Common causes of AKI include systemic inflammatory process, decreased kidney perfusion, obstruction of the urinary tract, and renal toxicity [10]. Among them, inflammation plays a key role. C-reactive protein (CRP), an essential major acute-phase protein, is the most commonly clinically used to reflect inflammation because the release of inflammatory cytokines causes its increased concentration and is associated with AKI mortality [11]. Albumin (ALB), the most abundant protein in plasma, is an indicator of human nutritional status and has also been reported to be associated with AKI [12]. Moreover, it has been proved that decreased ALB is associated with an inflammatory response [13]. Previous studies have demonstrated that higher CRP or lower ALB levels suggest a higher incidence of contrast agent-induced nephropathy [12, 14]. Furthermore, as a novel inflammatory prognostic score, CRP/albumin ratio (CAR) is helpful in predicting inflammatory diseases and cancers [15–18]. Therefore, we hypothesized that a CAR score could use to assess AKI mortality.

## 2. Methods

### 2.1. Population Selection Criteria

This is a single-center retrospective study. The included cases were patients admitted to the ICU of Shandong Provincial Hospital from January 2016 to November 2018 and diagnosed with AKI within 48 hours of ICU admission. Basal creatinine value was the lowest value measured after this admission. The AKI was determined by kidney disease's definition: Improved Global Outcomes (KDIGO) guidelines [19]. Patients meeting the following criteria were excluded: (1) c-reactive protein or albumin was not detected during ICU stay, (2) first-time ICU admission was less than 24 hours, (3) age was less than 18 years, and (4) missing value > 5%.

### 2.2. Data Extraction

Baseline demographic information, vital signs, routine laboratory parameters, complications, and other data were extracted from Shandong Provincial Hospital's electronic medical record system. Patient baseline demographic information and vital signs, including age, sex, mean arterial pressure (MAP), respiratory rate, heart rate, and temperature, were extracted. Complications include hypertension, coronary artery disease (CAD), kidney disease, and cancer. Routine laboratory parameters include CRP, ALB, urea nitrogen (BUN), creatinine, sodium, potassium, chloride, red blood cells (RBC), white blood cells (WBC), platelets, glucose, hematocrit, hemoglobin, mean corpuscular volume (MCV), triglycerides, total bilirubin (TBIL), red cell distribution width (RDW), and *β*2-microglobulin (BMG). The above records are measured within 48 hours of admission to ICU. Other extracted data included the AKI stage, AKI recovery, surgical grade, length of stay in the ICU, and whether the death occurred in the hospital. The state of renal function recovery was determined according to the last creatinine value before discharge. The last creatinine value ≤ 125% of base creatinine value was defined as recovery from AKI; otherwise, it is not recovered [20]. Two years after discharge, the included patients were followed up by telephone interviews to determine the two-year survival rate. The end of the observation period was November 2020, or loss to follow-up. Sequential organ failure assessment (SOFA) score [21] and acute physiological and chronic health score II (APACHE II) [22] were also performed for each patient.

### 2.3. Statistical Analysis

CAR tertiles stratified the clinical characteristics of all included cases. Continuous variables are presented as means ± SD or median (25th–75th percentile), and categorical data are described as numbers and percentages. The difference between the model development CAR tertiles groups was compared using Chi-squared tests for categorical variables and one-way analysis of variance (ANOVA) for continuous data. The variables with a skewed distribution used the Kruskal-Wallis test to compare. We performed multiple logistic regression analyses to determine the association between hospital mortality and 2-year mortality in CAR and AKI patients. We represented the odds ratio (OR) and 95% confidence interval (CI). We construct two multiple regression models to identify a statistical significant correlation between CAR and mortality; CAR's first tertile was used as the reference group. These confounding factors were selected based on a change in influence estimated at over 10% or the *P* values of regression coefficients <0.1 [23]. In model I, gender and age were adjusted as covariates. We adjusted for gender, age, respiratory rate, temperature, CAD, glucose, triglycerides, and surgical grade in model II. We performed a stratified analysis to assess whether the effects of CAR were consistent across subgroups classified by respiratory rate, temperature, hypertension, CAD, BUN, creatinine, sodium, potassium, WBC, RBC, glucose, hematocrit, hemoglobin, MCV, triglycerides, TBIL, RDW, BMG, recover from AKI or not, length of ICU stay, and surgical grade.

Furthermore, the generalized additive model was generated to measure the independent relationship between CAR and mortality, with adjustment for potential confounders: gender, age, respiratory rate, temperature, CAD, glucose, triglycerides, and surgical grade. The relationship between CAR and mortality was represented by a smooth curve and analyzed by the Chi-square test. *P* < 0.05 was considered statistically significant. The data has been analyzed using Empower Stats (http://www.empowerstats.com, X&Y solutions, Inc. Boston MA) and R software version 3.6.1 (https://www.r-project.org).

## 3. Results

### 3.1. Population Characteristics

According to the exclusion criteria, a total of 580 severe patients with AKI were eligible and included in this analysis (Figure 1). Based on CAR tertiles, the patients' population characteristics were described hierarchically and shown in Table 1. There were 193 patients in the low-CAR group (CAR < 0.21), 191 patients in the mid-CAR group (CAR ≥ 0.21, <2.54), and 196 patients in the high-CAR group (CAR ≥ 2.54). This subject included 371 (63.9%) men and 209 (36.1%) women. Patients in the high-CAR group had a higher proportion of older people and males and were more likely to suffer from hypertension and coronary heart disease. They also had lower hematocrit, hemoglobin, RBC level, and lower recovery rate. Moreover, these patients had a higher respiratory rate, heart rate, BUN, creatinine, WBC, glucose, triglycerides, TBIL, RDW, BMG, AKI stage, and surgical grade. Finally, they also had longer ICU stays, higher SOFA and APACHE II scores, and higher mortality than those in the low-CAR group.

### 3.2. CAR Is Associated with Clinical Prognosis

A higher CAR level was associated with higher in-hospital mortality and 2-year all-cause mortality in AKI patients admitted to ICU (Table 2). In model I, adjusted for gender and age, and compared with the low-CAR group (CAR < 0.21), the high-CAR group (CAR ≥ 16.43) adjusted ORs (95% CIs) of in-hospital mortality and 2-year all-cause mortality were 3.15 (1.90, 5.20) and 3.40 (2.00, 5.78), respectively. In model II, we adjusted for more confounders. We found that CAR remained an independent risk factor for increased in-hospital mortality and 2-year all-cause mortality in critically ill patients with AKI (the high-CAR group versus the low-CAR group: adjusted ORs, 95% CIs, *P* trends: 2.97, 1.70-5.17, <0.0001; 3.03, 1.68-5.47, 0.0002) (Table 2).

After adjusting for confounders, we found a linear relationship between CAR and in-hospital mortality, and the risk of in-hospital mortality of critically ill patients with AKI raised with the increase of CAR (*P* < 0.0001) (Figure 2(a)). Meanwhile, a similar trend was observed in 2-year mortality (*P* = 0.0043) (Figure 2(b)).

### 3.3. Subgroup Analyses

We performed a stratified analysis to determine that higher CAR levels in each subgroup were consistent with increased in-hospital mortality in patients admitted to ICU with AKI (Table 3). In female patients (OR, 5.4; 95% CI, 2.1 to 13.9) or who have undergone level 4 surgery (OR, 7.8; 95% CI, 2.9 to 21.0), the higher the CAR level, the higher risk of the hospital mortality. Similarly, patients with high values of glucose (OR, 6.1; 95% CI, 2.2 to 17.0), TBIL (OR, 6.5; 95% CI, 2.3 to 18.4), and WBC (OR, 9.6; 95% CI, 2.2 to 42.9) were at higher risk with increased CAR. The table also shows that in-hospital mortality increases with the increase of CAR regardless of recovery from AKI or not.

## 4. Discussion

In conclusion, we established that a higher level of CAR was associated with a significantly increased risk of in-hospital mortality and 2-year all-cause mortality in patients who developed AKI after admission to the ICU. After adjusting for gender and age, or for more covariates, this significant correlation remains. Both CRP and ALB can be controlled by various clinical treatment methods. The findings of this study may help clinicians to take early treatment measures to reduce the mortality of critically ill patients with AKI.

Although the pathogenesis of AKI remains unclear, previous studies have shown that AKI is associated with high circulating levels of inflammatory mediators [24]. The inflammatory mediators are related to the prognosis of AKI, including CRP, ALB, lymphocytes, tumor necrosis factor receptor I (TNF-R-I), TNF-R-II, neutrophils, platelets, interleukin (IL) 1, IL-6, IL-10, and RDW [25–29]. Among them, CRP, as a significant marker of the inflammatory response, can reduce the expression of endothelial nitric oxide synthase (eNOS) and mRNA stability, promote the expression of endothelial lox-1, stimulate ROS production, and increase endothelial cell apoptosis, and thus promote endothelial dysfunction, which is the main factor of AKI [30]. Tang et al. [31] reported that the role of CRP had been gradually recognized as a factor promoting the occurrence and progression of AKI by preventing the repair and proliferation of damaged renal tubular epithelial cells, increasing inflammatory response, and promoting the fibrosis of damaged renal tissue in recent years. ALB, a protein synthesized in the liver, is generally regarded as a nutritional status marker and has several vital functions, including carrying poorly water-soluble molecules, regulating osmotic pressure, antioxidants, and anti-inflammatory effects, which has a protective effect on the kidneys [32, 33]. Hypoalbuminemia makes the body unable to remove toxic substances effectively and leads to decreased vascular volume followed by renal hypoperfusion, and both of them will cause kidney damage [34]. Low ALB serum levels may be associated with systemic inflammatory response syndrome. Several studies have shown that hypoproteinemia can increase the morbidity and mortality of AKI in critically ill patients [35, 36].

Therefore, we introduced the concept of CAR, which reflects the combination of inflammation and nutrition. CAR is associated with the prognosis of many diseases, including various cancers (e.g., advanced nonsmall-cell lung cancer and nasopharyngeal carcinoma), inflammatory diseases (e.g., acute pancreatitis and acute severe ulcerative colitis), and cardiovascular diseases [15–18, 37–39]. According to the above mechanism and previous reports, our results were reasonable.

There were some pitfalls and limitations in this study. First, this is an observational, retrospective, single-center study, possibly introducing selection bias. Second, we only calculated the CAR when the patient was admitted to the ICU and did not record the changes in laboratory results during the ICU period, which may cause inaccuracy of the products. Third, attempts have been made to control the study's confounding biases using multivariate analysis techniques, but some unknown confounding factors or information failed to collect. Fourth, we did not have the exact death time of the included cases to do the K-M survival curve. Finally, a retrospective study has some inevitable defects due to its nature; therefore, prospective, multicentered studies should be performed to corroborate these findings.

## 5. Conclusions

We analyzed the clinical data of 580 patients in the electronic medical record system of Shandong Provincial Hospital. Our results show that higher CAR was associated with an increased risk of in-hospital mortality and 2-year all-cause mortality in critically ill patients with AKI. However, further prospective multicenter studies are still needed to confirm our findings.

## Figures and Tables

**Figure 1:** Illustration of exclusion criteria as utilized to select the final 580 patients.

**Figure 2:** Association between CAR and in-hospital mortality (a) and 2-year all-cause mortality (b) in critically ill patients with AKI. A linear association between CAR and mortality was found in a generalized additive model (GAM). Solid red line represents the smooth curve fit between variables. Blue bands represent the 95% of confidence interval from the fit. All adjusted for age, gender, respiratory rate, temperature, CAD, glucose, triglycerides, and surgical grade.

**Table 1:** Characteristics of the study patients according to CAR.

Characteristics	CRP to albumin ratio			*P* value
	0-0.2 (*n* = 193)	0.21-2.53 (*n* = 191)	2.54-16.43 (*n* = 196)	
Age (years)	57.3 ± 14.9	56.1 ± 17.5	62.6 ± 15.1	<0.001
Gender (*n* (%))				0.022
Male	111 (57.5%)	121 (63.4%)	139 (70.9%)	
Female	82 (42.5%)	70 (36.6%)	57 (29.1%)	
CAR	0.0 (0.0-0.1)	0.9 (0.4-1.7)	5.1 (3.7-7.6)	<0.001
Respiratory rate (beats/minute)	20.3 ± 7.6	20.9 ± 7.2	21.5 ± 8.0	<0.001
Temperature (°C)	36.6 ± 0.6	36.6 ± 0.7	36.7 ± 0.8	0.036
Heart rate (beats/minute)	91.2 ± 20.6	95.4 ± 25.4	96.5 ± 26.5	0.266
MAP (mmHg)	96.8 ± 21.3	92.4 ± 19.6	92.9 ± 21.8	0.08
Laboratory parameters				
Albumin (g/L)	36.1 ± 6.7	32.9 ± 7.4	28.4 ± 6.6	<0.001
CRP (mg/L)	1.5 (0.7-2.9)	5.9 (12.5-54.7)	151.4 (110.5-205.0)	<0.001
BUN (mmol/L)	6.1 (4.6-9.0)	7.6 (5.2-12.6)	8.0 (5.3-12.5)	<0.001
Chloride (mmol/L)	105.3 ± 4.9	105.4 ± 33.8	103.1 ± 10.9	0.005
Creatinine (*μ*mol/L)	154.4 (118.0-211.9)	179.5 (124.4-254.8)	182.8 (131.0-252.0)	0.029
Glucose (mmol/L)	5.4 (4.9-7.0)	6.4 (5.2-8.5)	7.0 (5.3-10.0)	<0.001
Potassium (mmol/L)	4.3 ± 0.6	4.1 ± 0.6	4.1 ± 0.7	0.017
Sodium (mmol/L)	140.1 ± 3.4	138.4 ± 5.7	139.1 ± 11.8	0.001
Triglycerides (mmol/L)	1.2 (0.9-1.8)	1.3 (0.9-1.9)	1.4 (0.9-2.1)	0.151
BMG (mg/L)	2.5 (1.9-3.5)	3.0 (2.2-5.1)	3.0 (2.2-5.6)	<0.001
Hematocrit (%)	37.6 ± 6.8	34.8 ± 8.2	35.4 ± 8.4	0.002
Hemoglobin (g/L)	126.1 ± 25.1	115.4 ± 28.8	117.8 ± 29.1	<0.001
MCV (fL)	90.3 ± 8.1	89.3 ± 9.1	90.6 ± 10.6	0.017
Platelets (10^9^/L)	176.0 (135.0-227.0)	187.0 (116.0-232.0)	181.0 (103.5-248.0)	0.896
RBC (10^12^/L)	4.2 ± 0.8	3.9 ± 0.9	3.9 ± 0.9	0.002
RDW (%)	13.8 ± 1.8	14.3 ± 1.9	14.3 ± 2.4	0.005
WBC (10^9^/L)	6.4 (5.1-8.9)	8.9 (5.9-12.2)	9.5 (6.5-13.9)	<0.001
TBIL (*μ*mol/L)	13.9 (10.2-19.7)	15.2 (10.8-22.5)	15.9 (10.9-26.5)	0.047
Scoring systems				
APACHE II	12.0 (8.0-17.0)	15.0 (10.0-20.0)	18.0 (12.0-23.0)	<0.001
SOFA	4.0 (2.0-5.0)	5.0 (3.0-7.5)	5.0 (3.0-8.0)	<0.001
Comorbidities (*n* (%))				
Hypertension	93 (48.2%)	73 (38.2%)	111 (56.6%)	0.001
Diabetes	43 (22.3%)	32 (16.8%)	37 (18.9%)	0.383
Coronary artery disease	23 (11.9%)	16 (8.4%)	37 (18.9%)	0.008
Acute cerebral infarction	26 (13.5%)	15 (7.9%)	27 (13.8%)	0.127
Cancer	3 (1.6%)	4 (2.1%)	13 (6.6%)	0.011
Surgical grade (*n* (%))				<0.001
No surgery or grade 1	51 (26.4%)	81 (42.4%)	66 (33.7%)	
Grade 2	44 (22.8%)	17 (8.9%)	15 (7.7%)	
Grade 3	15 (7.8%)	11 (5.8%)	10 (5.1%)	
Grade 4	83 (43.0%)	82 (42.9%)	105 (53.6%)	
AKI stage (*n* (%))				0.037
Stage 1	138 (71.5%)	115 (60.2%)	115 (58.7%)	
Stage 2	33 (17.1%)	55 (28.8%)	56 (28.6%)	
Stage 3	22 (11.4%)	21 (11.0%)	25 (12.8%)	
ICU LOS (days)	4.0 (2.0-9.0)	7.0 (3.5-12.0)	9.0 (4.0-15.0)	<0.001
Recovery from AKI (*n* (%))	141 (73.1%)	129 (66.8%)	106 (54.6%)	<0.001
Hospital mortality (*n* (%))	28 (14.5%)	43 (22.5%)	75 (38.3%)	<0.001
2-year mortality (*n* (%))	46 (36.2%)	69 (57.5%)	101 (69.7%)	<0.001

CAR: C-reactive protein-to-albumin ratio; CRP: C-reactive protein; MAP: mean arterial pressure; BUN: blood urea nitrogen; BMG: *β*2-microglobulin; MCV: mean corpuscular volume; RBC: red blood cells; RDW: red cell distribution width; WBC: white blood cells; TBIL: total bilirubin; SOFA: sequential organ failure assessment; APACHE II: acute physiological and chronic health score II; AKI: acute kidney injury; ICU: intensive care unit; LOS: length of stay.

**Table 2:** Relationship between CAR and mortality.

CAR	Nonadjusted		Model I		Model II	
	OR (95% CIs)	*P* value	OR (95% CIs)	*P* value	OR (95% CIs)	*P* value
Hospital mortality						
Per 1 sd change	1.71 (1.42, 2.04)	<0.0001	1.59 (1.32, 1.91)	<0.0001	1.73 (1.40, 2.13)	<0.0001
Tertiles						
0-0.2	1.0 (ref)		1.0 (ref)		1.0 (ref)	
0.21-2.53	1.71 (1.01, 2.89)	0.0448	1.71 (1.00, 2.91)	0.0496	1.57 (0.88, 2.78)	0.1240
2.54-16.43	3.65 (2.23, 5.98)	<0.0001	3.15 (1.90, 5.20)	<0.0001	2.97 (1.70, 5.17)	0.0001
*P* trend	<0.0001		<0.0001		<0.0001	
2-year mortality						
Per 1 sd change	1.88 (1.47, 2.39)	<0.0001	1.69 (1.33, 2.16)	<0.0001	1.76 (1.35, 2.29)	<0.0001
Tertiles						
0-0.2	1.0 (ref)		1.0 (ref)		1.0 (ref)	
0.21-2.53	2.38 (1.43, 3.97)	0.0009	2.53 (1.47, 4.36)	0.0008	2.26 (1.26, 4.07)	0.0063
2.54-16.43	4.04 (2.44, 6.71)	<0.0001	3.40 (2.00, 5.78)	<0.0001	3.03 (1.68, 5.47)	0.0002
*P* trend	<0.001		0.0002		0.0021	

OR: odds ratio; CI: confidence interval. Adjust I model, adjusted for age and gender. Adjust II model, adjust for age, gender, respiratory rate, temperature, CAD, glucose, triglycerides, and surgical grade.

**Table 3:** Effect size of CAR on hospital mortality in prespecified and exploratory subgroups in each subgroup.

	CRP to albumin ratio (CAR)				
	0-0.2	0.21-2.53		2.54-16.43	
		OR (95% CIs)	*P* trend	OR (95% CIs)	*P* trend
Gender					
Male	1.0 (ref)	1.5 (0.8, 2.8)	0.223	2.9 (1.6, 5.2)	<0.001
Female	1.0 (ref)	2.2 (0.8, 6.0)	0.116	5.4 (2.1, 13.9)	<0.001
Recovery from AKI					
Yes	1.0 (ref)	1.3 (0.7, 2.4)	0.414	2.3 (1.3, 4.3)	0.007
No	1.0 (ref)	3.7 (1.3, 10.7)	0.017	8.2 (3.0, 22.6)	<0.001
Age (year)					
<52	1.0 (ref)	1.7 (0.6, 4.8)	0.326	3.5 (1.2, 10.2)	0.019
≥53, <66	1.0 (ref)	2.2 (0.8, 5.8)	0.110	4.6 (1.9, 10.9)	<0.001
≥67	1.0 (ref)	1.4 (0.6, 3.2)	0.418	2.5 (1.2, 5.3)	0.017
Respiratory rate (beats/minute)					
<18	1.0 (ref)	3.2 (0.7, 14.5)	0.133	8.2 (2.2, 30.9)	0.002
≥18, <20	1.0 (ref)	2.1 (0.7, 5.9)	0.158	3.4 (1.1, 10.0)	0.028
≥20	1.0 (ref)	1.2 (0.6, 2.4)	0.542	2.8 (1.5, 5.3)	0.001
BUN (mmol/L)					
<5.6	1.0 (ref)	1.7 (0.7, 4.3)	0.230	3.9 (1.7, 9.1)	0.001
≥5.6, <9.4	1.0 (ref)	1.8 (0.7, 4.6)	0.206	3.9 (1.7, 9.4)	0.002
≥9.4	1.0 (ref)	1.4 (0.6, 3.6)	0.474	2.8 (1.2, 6.9)	0.022
Creatinine (*μ*mol/L)					
<140.09	1.0 (ref)	1.6 (0.6, 4.3)	0.388	6.1 (2.5, 15.2)	<0.001
≥140.09, <207	1.0 (ref)	2.4 (1.0, 5.9)	0.055	3.9 (1.7, 9.2)	0.002
≥207	1.0 (ref)	1.1 (0.5, 2.6)	0.803	2.0 (0.9, 4.5)	0.109
Sodium (mmol/L)					
<138	1.0 (ref)	1.4 (0.5, 3.8)	0.509	3.1 (1.1, 8.3)	0.028
≥138, <141	1.0 (ref)	1.8 (0.7, 4.9)	0.226	3.5 (1.4, 8.9)	0.009
≥141	1.0 (ref)	1.4 (0.6, 3.2)	0.478	3.4 (1.6, 7.2)	<0.001
Potassium (mmol/L)					
<3.9	1.0 (ref)	2.4 (0.7, 8.1)	0.144	6.3 (2.0, 19.7)	0.001
≥3.9, <4.3	1.0 (ref)	1.6 (0.7, 3.7)	0.267	2.8 (1.2, 6.4)	0.015
≥4.3	1.0 (ref)	1.7 (0.7, 3.9)	0.236	3.4 (1.6, 7.6)	0.002
RBC (10^12^/L)					
<3.71	1.0 (ref)	2.2 (0.7, 7.4)	0.180	5.2 (1.7, 16.2)	0.004
≥3.71, <4.5	1.0 (ref)	1.5 (0.6, 3.5)	0.360	3.5 (1.6, 8.0)	0.002
≥4.5	1.0 (ref)	2.3 (0.9, 5.9)	0.074	3.9 (1.6, 9.6)	0.002
WBC (10^9^/L)					
<6.17	1.0 (ref)	1.8 (0.7, 4.2)	0.203	4.9 (2.1, 11.4)	<0.001
≥6.17, <10.36	1.0 (ref)	1.9 (0.8, 4.5)	0.150	2.5 (1.1, 5.8)	0.030
≥10.36	1.0 (ref)	3.7 (0.8, 17.3)	0.098	9.6 (2.2, 42.9)	0.003
Glucose (mmol/L)					
<5.35	1.0 (ref)	2.0 (0.9, 4.7)	0.099	1.9 (0.8, 4.4)	0.125
≥5.35, <7.65	1.0 (ref)	1.1 (0.4, 2.9)	0.776	3.2 (1.3, 8.0)	0.011
≥7.65	1.0 (ref)	2.5 (0.8, 7.5)	0.098	6.1 (2.2, 17.0)	<0.001
Hematocrit (%)					
<33.4	1.0 (ref)	2.0 (0.7, 6.1)	0.203	4.2 (1.5, 11.8)	0.007
≥33.4, <40.2	1.0 (ref)	1.4 (0.6, 3.3)	0.398	3.1 (1.3, 7.0)	0.008
≥40.2	1.0 (ref)	2.5 (0.9, 6.6)	0.067	5.6 (2.3, 13.6)	<0.001
Hemoglobin (g/L)					
<110	1.0 (ref)	2.8 (0.9, 9.1)	0.081	4.2 (1.4, 13.2)	0.013
≥110, <136	1.0 (ref)	1.1 (0.5, 2.6)	0.754	3.2 (1.5, 7.1)	0.004
≥136	1.0 (ref)	2.7 (1.0, 7.4)	0.052	6.7 (2.7, 17.1)	<0.001
MCV (fL)					
<87.3	1.0 (ref)	1.8 (0.7, 4.6)	0.253	3.1 (1.2, 8.1)	0.023
≥87.3, <92.1	1.0 (ref)	1.7 (0.7, 4.0)	0.240	4.2 (1.8, 9.5)	<0.001
≥92.1	1.0 (ref)	2.4 (0.9, 6.7)	0.097	5.2 (2.1, 12.8)	<0.001
Triglycerides (mmol/L)					
<1.04	1.0 (ref)	2.8 (0.9, 8.3)	0.065	9.9 (3.5, 28.0)	<0.001
≥1.04, <1.68	1.0 (ref)	1.3 (0.6, 3.0)	0.483	1.5 (0.6, 3.3)	0.371
≥1.68	1.0 (ref)	1.7 (0.6, 4.7)	0.328	4.0 (1.6, 10.1)	0.004
TBIL (*μ*mol/L)					
<11.9	1.0 (ref)	1.0 (0.4, 2.4)	0.956	1.7 (0.7, 3.8)	0.220
≥11.9, <19.3	1.0 (ref)	2.0 (0.8, 4.9)	0.111	4.5 (1.9, 10.6)	<0.001
≥19.3	1.0 (ref)	2.5 (0.8, 7.6)	0.095	6.5 (2.3, 18.4)	<0.001
RDW (%)					
<13.2	1.0 (ref)	2.6 (1.0, 6.9)	0.059	4.7 (1.9, 11.3)	<0.001
≥13.2, <14.2	1.0 (ref)	1.5 (0.6, 3.9)	0.347	4.2 (1.8, 10.2)	0.001
≥14.2	1.0 (ref)	1.7 (0.7, 4.5)	0.269	3.4 (1.3, 8.5)	0.010
BMG (mg/L)					
<2.31	1.0 (ref)	2.3 (1.0, 5.5)	0.065	3.9 (1.7, 9.0)	0.001
≥2.31, <3.69	1.0 (ref)	1.6 (0.7, 4.0)	0.288	3.5 (1.5, 8.2)	0.004
≥3.69	1.0 (ref)	1.3 (0.5, 3.5)	0.611	3.2 (1.3, 8.2)	0.013
ICU LOS (days)					
<4	1.0 (ref)	2.9 (1.1, 7.7)	0.035	3.7 (1.4, 10.0)	0.010
≥4, <10	1.0 (ref)	2.7 (1.1, 6.9)	0.039	5.1 (2.0, 12.9)	<0.001
≥10	1.0 (ref)	0.6 (0.3, 1.5)	0.303	1.9 (0.9, 4.1)	0.096
Surgical grade					
No surgery or grade 1	1.0 (ref)	1.7 (0.8, 3.9)	0.192	4.1 (1.8, 9.4)	<0.001
Grade 2	1.0 (ref)	0.0 (0.0, Inf)	0.991	1.4 (0.4, 5.5)	0.617
Grade 3	1.0 (ref)	0.9 (0.1, 6.5)	0.908	0.4 (0.0, 5.0)	0.512
Grade 4	1.0 (ref)	3.5 (1.2, 10.1)	0.021	7.8 (2.9, 21.0)	<0.001

CRP: C-reactive protein; BUN: blood urea nitrogen; RBC: red blood cells; WBC: white blood cell; MCV: mean corpuscular volume; TBIL: total bilirubin; RDW: red cell distribution width; BMG: *β*2-microglobulin; ICU: intensive care unit; LOS: length of stay.

## Data Availability

The data of this study are all from the electronic medical record system of Shandong Provincial Hospital, and source data can be obtained from the corresponding author Yong Wang if reasonably requested.
